The article "Green Synthesis of Silver Nanoparticles Using Thespesia populnea Bark Extract for Efficient Removal of Methylene Blue (MB) Degradation via Photocatalysis with Antimicrobial Activity and for Anticancer Activity" was published in 2022. Journal: Bioinorg Chem Appl.

# Green Synthesis of Silver Nanoparticles Using *Thespesia populnea* Bark Extract for Efficient Removal of Methylene Blue (MB) Degradation via Photocatalysis with Antimicrobial Activity and for Anticancer Activity

**DOI:** 10.1155/2022/7268273

**Published:** 2022-06-30

**Authors:** Muhammad Yahya Tahir, Awais Ahmad, Asma A. Alothman, Mohammed Sheikh Saleh Mushab, Shafaqat Ali

**Affiliations:** ^1^Department of Environmental Science and Engineering, Government College University Faisalabad, Faisalabad 38000, Pakistan; ^2^Departamento de Quimica Organica, Universidad de Cordoba, Edificio Marie Curie (C-3), Ctra Nnal IV-A, Km 396, Cordoba E14014, Spain; ^3^Department of Chemistry, College of Science, King Saud University, Riyadh 11451, Saudi Arabia; ^4^Department of Biological Sciences and Technology, China Medical University, Taichung 40402, Taiwan

## Abstract

The green synthesis method was used to effectively fabricate Ag-NPs by using *Thespesia populnea* bark extract. The structural, morphological, elemental composition, and optical properties of as-synthesized Ag-NPs were characterized by powder X-ray diffraction (P-XRD), Fourier transform infrared spectroscopy (FTIR), scanning electron microscopy (SEM), energy-dispersive X-ray spectroscopy (EDAX), transmission electron microscopy (TEM), and UV-Vis spectroscopy. Their photocatalytic efficiency as a photocatalyst was examined by degradation of methylene blue (MB) dye under direct sunlight irradiation. After 120 minutes of sunlight irradiation, Ag-NPs show photocatalytic degradation efficiency (DE percent) of 92%. The hydroxyl and superoxide radicals were found to be responsible for biodegradation. To the best of our acquaintance, this is the first research to use Ag-NPs as a photocatalyst for the efficient degradation of MB dye and its antimicrobial activity by using *Thespesia populnea* bark extract. The cytotoxic viability against SK-MEL cell line with a median inhibitory concentration (IC_50_) of 45 *μ*L/mg proved its potent anticancer property. Based on the findings, the study revealed the significance of as-synthesized green Ag-NPs over other physically/chemically prepared Ag-NPs.

## 1. Introduction

Water pollution has become one of the most severe environmental concerns caused by the disposal of harmful and toxic contaminants such as organic dyes and heavy metal ions in recent decades. Heavy metals and dyes are mainly merged in the ecological system through industrial effluent streams and pose serious threats to human health [1]. Dyes are the most commonly used substances in textile and cosmetic industries, and they are released into the environment directly. Their accumulation has been increased due to increased industrial operations, technological progress, and ineffective preventive measures [2]. The carcinogenic nature of dyes, low biodegradability, and half-life of more than 2000 hours under sunlight irradiation have urged researchers to invent a constant solution [3]. Therefore, a lot of research work has been reported to develop effective environmental remediation technologies. Several approaches have been devised, for example, electrochemical oxidation, membrane filtration, biodegradation, ozonation, and adsorption. However, nanotechnology is a growing area of attention since nanoparticles (NPs) have applications in almost every field of life [4]. Among various approaches to remediate the environment, photocatalysis via nanostructured semiconductors has become one of the steadiest research topics of nanoscience and nanotechnology. This approach has engrossed attention for its ability to remove organic pollutants from the environment [5]. Noble metal nanoparticles have gained more attention than other metal nanoparticles due to their high surface-to-volume ratio and small size [6].

In general, recent years have raised a new trend to synthesize NPs through biological ways. Nanoparticles synthesized from biological sources such as plant extracts are eco-friendly, nontoxic, cost-effective, and highly effectual and can also be used in drug delivery; on the other hand, chemically synthesized NPs can be hazardous and toxic [7, 8]. Biologically synthesized NPs are devised by sustainable and green methods and are now widely used in pharmaceutical industries due to their remarkable properties [9]. Despite the fact that plant extracts include various secondary metabolites with significant reducing potential, they can be used as reducing and stabilizing agents to synthesize green NPs [10]. Green synthesis of NPs by using plant extracts is an advanced as well as a cost-effective approach [11]. In this regard, silver nanoparticles (Ag-NPs) possess remarkable antimicrobial, chemical, structural, and optical properties among other metal nanoparticles [12]. Ag-NPs synthesized using plant extracts can be used as nanocatalysts [13, 14]. Various green synthesis routes as well as other biological methods for the synthesis of Ag-NPs by using plant extracts and microorganisms are reported to date. Additionally, Ag-NPs synthesized by green approaches possess several important properties such as antibacterial, antioxidant, medical diagnostics, therapeutic, and cytotoxic [10]. In the present study, we have prepared Ag-NPs using *Thespesia populnea* bark extract [15, 16].

In this context, plants are considered one of the most communal, effective, efficient, reasonable, and eco-friendly sources of nanomaterials [14]. Plant extracts contain various secondary metabolites, which play an important role in revitalizing the metal ions during the synthesis of NPs by an eco-friendly reaction [15]. *Thespesia populnea* (family *Malvaceae*) is a fast-growing tree, occurring naturally in tropical areas, coastal woods, and gardens. Its bark, root, and fruits are used in Ayurveda to cure diabetes, dysentery, cholera, and haemorrhoids [17]. Its bark has been described in the Siddha system of medicine as being used to reduce swelling and oedema [18]. The bark and flowers possess hepatoprotective, antioxidant, and anti-inflammatory properties. Different phytochemicals, for example, glucose, protein, tannins, phenol, flavonoids, terpenoids, saponins, and gums, have been found in different parts of tree [19, 20].

However, to the best of our knowledge, the green synthesis of Ag-NPs using *Thespesia populnea* bark extract has not been reported yet. Hence, in the light of the aforementioned factors and the prerequisite to developing a meaningful and alternate source for the degradation of MB dye, the present work was designed to synthesize Ag-NPs by using *Thespesia populnea* extract. Furthermore, the current study also aimed to assess potential antimicrobial and anticancer activity of as-prepared NPs for enhanced environmental applications.

## 2. Materials and Methods

### 2.1. Materials

All the chemicals and reagents used in this study were of high-quality analytical grade. Silver nitrate (AgNO_3_, ≥99%) was purchased from Sigma Aldrich and used in the experiment without any further purification. Deionized water was freshly prepared and used during the whole experiment.

### 2.2. Green Synthesis of Silver Nanoparticles from *Thespesia populnea* Bark Extract

Silver nanoparticles (Ag-NPs) were synthesized by using *Thespesia populnea* bark extract. The synthesis of Ag-NPs was carried out by following the protocol reported by Aravind et al. [21] with slight modification. Prior to synthesis, bark extract was synthesized, and it served as a capping agent. A solution of silver nitrate (1 M) was prepared in 90 ml of deionized water. 20 ml of bark extract was dissolved in prepared AgNO_3_ solution, and the solution was stirred at room temperature for 30 minutes. In order to purify the prepared solution, it was washed three times with double-distilled water and centrifuged at 4000 rpm for 10 minutes. The obtained sample was dried in a hot air oven at 100°C for 1 hour.  Figure 1 shows a schematic diagram for the synthesis of Ag-NPs.

### 2.3. Characterization of Silver Nanoparticles

The XRD patterns of as-prepared NPs were analysed by X-ray diffraction (PAN analytical X'PERT PRO diffractometer). The UV-visible spectra were gained by UV-visible absorbance spectrophotometer (Shimadzu Elico-169 PC scanning double beam UV-visible spectrophotometer). The basic morphology of prepared nanoparticles, along with their size, was determined by Scanning Electron Microscope with Energy-Dispersive Spectra (EVO18 (CARL ZEISS)), Quantax 200 with X Flash® 6130, and Transmission Electron Microscopic (JEOL JEM 2100). The functional groups and phytochemicals involved in degradation were categorized by Fourier Transform Infrared Spectrum (Perkin Elmer RXI spectrometer).

### 2.4. Antibacterial Activity

The antibacterial activity of green synthesized nanoparticles against *E. coli* and *S. aureus* was analysed by means of disc diffusion assay. The bacterial cultures were grown in a nutrient medium. The overnight grown cultures of *E. coli* and *S. aureus* were swabbed uniformly on nutrient agar plates. Sterile paper discs (3 mm) were prepared containing 50 *μ*g/ml of as-prepared silver nanoparticles. These discs were added to the prepared plates and incubated at 37°C for 24 h. After incubation of 24 h, zones of inhibition were observed.

### 2.5. Photocatalytic Activity

The photocatalytic activity of as-prepared photocatalyst (Ag-NPs) for the degradation of MB dye was detected under solar irradiation. The Ag-NPs were disseminated in 100 mL of an aqueous solution of MB dye. Prior to irradiation, the synthesized solution was ultrasonicated and agitated for 30 minutes in a darkroom in order to analyse the adsorption/desorption conditions. Then, the solution was irradiated with direct sunlight while being magnetically stirred. After every 10 minutes, 5 ml of suspension was taken, centrifuged at 3000 rpm for 10 minutes, and finally kept at 37°C. The photodegradation of dye was monitored by UV-Vis spectrophotometer at different time intervals.

### 2.6. Anticancer Activity

#### 2.6.1. Cell Cytotoxicity (MTT) Assay

SK-MEL cell lines were cultured at 37°C and 5% CO_2_ for 24 hours in an incubator. Then, the cells were seeded on 96-well plates, approximately 2500 cells/well. The cytotoxicity of green synthesized Ag-NPs on SK-MEL cells was determined by MTT assay. The test samples were prepared in DMEM media (100 mg/mL) and cleansed by using a Millipore syringe filter of 0.2 m. The samples were further diluted by DMEM medium, and final concentrations of 12.5 and 50 g/mL, respectively, were obtained. The prepared and diluted samples were added to the cultured cell wells. The plates were then incubated for another 24 h after being treated with the test samples. The wells without containing cell sample were taken as control. The medium was removed from the sample after incubation. Then, the wells were filled with 100 mL of 0.5 mg/mL MTT solution in PBS. The plates were then incubated for another 2 h to allow the formation of formazan crystals. The formazan crystals were further dissolved in 100 mL of 100% dimethyl sulphoxide (DMSO) and applied to each well. These crystals were observed at 570 nm by a microplate reader.

All the tests were executed in triplicate, and average data were analysed. The cytotoxic effect of nanoparticles on the cells was calculated as the percentage viability of the cells by using the following formula:

(1) $$\begin{array}{c} \text{Percentage of cell viability}=\frac{\text{Average absorbance of treated}}{\text{Average absorbance of control}}\times 100. \end{array}$$

## 3. Results and Discussion

### 3.1. XRD Analysis

Figure 2 shows the XRD pattern of Ag-NPs by using *Thespesia populnea* bark extract. XRD pattern showed diffraction peaks at 32.4^o^, 44.6^o^, 64.2^o^, and 77^o^, which can be corresponded to similar Braggs reflection planes of (111), (200), (220), and (311), respectively. The observed XRD pattern was well-matched with standard JCPDS No. 04–0783 [22]. The as-prepared Ag-NPs have a face-centred cubic structure. At the same time, additional peaks connected with standard Ag peaks can be attributed to the presence of phytochemicals extracted from *Thespesia populnea*, which might get capped on the surface of NPs [23, 24]. The width of the (111) Bragg's reflection was used to calculate the average size of the fabricated Ag-NPs by using the Debye–Scherer equation (2).

(2) $$\begin{array}{c} D=\frac{k\lambda }{\beta \text{Cos}\theta }, \end{array}$$

where *D* embodies the average crystallite size value (nm), *k* denotes Scherer's constant, *λ* represents the wavelength of X-ray, *β* is the full width half maximum, and *θ* is the angle of diffraction [25]. The average crystallite size was calculated to be 19.05 nm.

### 3.2. Fourier Transform Infrared Spectrum

FTIR analysis was used to detect the surface functional groups and their interaction, present in as-synthesized Ag-NPs. The pragmatic FTIR spectrum of as-prepared Ag-NPs is shown in Figure 3. The spectrum showed major absorption peaks of 3276, 2926, 1636, 1327, 1021, 810, and 512 cm^−1^, which can be assigned to O–H [26], C–H [27, 28], C–C, C–O, –C-O, -C-H (alkanes), and COO- stretching vibrations [29], respectively, signifying that the phytochemicals in the extract act as a capping agent, which bound to the Ag-NPs. According to FTIR analysis, the presence of phytochemicals, for example, amide group, an amino group, carboxyl group tannins, phenol, flavonoids, terpenoids, saponins, and polyphenolic compound in the *Thespesia populnea* bark extract, played a critical role in the reduction, capping, and stabilization of Ag-NPs [30]. FTIR also revealed that the bimolecular compounds are responsible for the reduction of Ag^+^ ions to Ag-NPs. The wide and asymmetric nature of the *C*=*C* stretching vibrations of adsorbed on the surface of Ag-NPs can be attributed to the reduction of Ag^+^to Ag^0^ state [31].

### 3.3. UV-Visible Spectroscopy

UV-Vis spectroscopy was used to inspect the optical characteristics of synthesized Ag-NPs. The absorption peak in the UV-Vis region in absorbance spectra confirmed the Ag-NPs (Figure 4). The detection of absorption peak is due to the Surface Plasmon Resonance (SPR) of silver NPs. Due to the excitation of surface plasmon, the Ag-NPs showed a strong absorption peak in the Vis region. Due to SPR, the reduction of AgNO_3_ to Ag-NPs was initially observed by detecting the change in colour of the mixture from colourless to brown [32]. Moreover, the SPR absorption band was detected due to the simultaneous oscillation of free conduction electrons of metal in resonance with a light wave. The particle size, dielectric medium, and chemical environment impact the absorption spectra. Ag-NPs fashioned a wide SPR band at 446 nm, indicating the production of NPs of different morphology [33]. The spike observed around 340 nm corresponds to the unabsorbed biomolecules present on the surface of Ag-NPs. The SPR bands of the produced colloids showed a blue shift in the reaction media [34]. The plasmon absorption peak is affected by particle size, shape, nucleophile, and electrophile adsorption on the particle surface.

A blue shift is usually linked to reduction in particle size or donation of electron density from the surface. The adsorption of the nucleophile on the surface of Ag-NPs augments the Fermi level by donating electron density to the particles [35, 36]. The lack of peaks in the higher wavelength area and the symmetric character of the SPR showed the absence of nanoparticle aggregation, verified by TEM. The optical stability of the nanoparticles was confirmed after four months. The Ag-NPs were stable after four months and had a typical absorption of ∼420–450 nm, within the Ag-NPs range, as shown in Figure 5.

### 3.4. Scanning Electron Microscope

Figure 6 shows SEM images of prepared Ag-NPs by using *Thespesia populnea* bark extract. The extract confined capping molecules such as chlorophyll, carotenoids, and anthocyanins, which combined with AgNO_3_ to form Ag nanoparticles. The size, shape, and morphology of as-fabricated Ag-NPs were studied by using SEM. The results revealed the spherical shape of Ag-NPs with 40–50 nm diameter. The synthesis of Ag-NPs is found to be influenced by various factors, including concentration of reducing agent, metal salt, and time. On the other hand, the stabilizing agents and modifiers played an essential role in regulating the form of particles by avoiding agglomeration [37, 38].

### 3.5. Elemental Dispersive Analyses Spectrum

The elemental composition of Ag-NPs obtained from green synthesis is shown in Figure 7. From the EDAX spectrum, Ag is considered the primary compound. EDS spectra confirmed the synthesis of Ag-NPs. EDS graph indicated the presence of certain elements, including silver (Ag), oxygen (O), and carbon (C), in the sample. The presence of 3 keV peaks proposed that Ag is present in the elemental form [39]. The undefined peaks correspond to untreated biomolecules present in the extract. The presence of carbon peak can be attributed to the presence of C–C, C–H, C–OH, *C*=*O*, and C–O–C.

### 3.6. Transmission Electron Microscope (TEM)

TEM images of as-fabricated Ag-NPs are shown in Figure 8. TEM image confirms the uniform distribution of monodispersive spherical Ag-NPs. The presence of uniformly scattered and symmetrically spherical NPs with an average size of 10 nm can be observed in the TEM images of Ag-NPs. The generation of spherical NPs can be attributed to the interaction between biomolecules present in the extract [40]. The twinned nanoparticles were detected by comparing the brightness of different sections of the particles, such as face-centred cubic (FCC) structured metallic nanocrystals, twinning, or the planar defect. Distinct surface energies exist for different crystal planes in noble metals' face-centred cubic lattice [41].

### 3.7. Photocatalytic Activity

Methylene blue (MB) dye was used as a reference pollutant dye to analyse the photocatalytic activity of as-fabricated Ag-NPs.  Figure 9(a) shows the MB dye photodegradation spectrum after 120 minutes under visible-light irradiation. The absorbance of light decreases steadily with time at 655 nm. Additionally, the absorption spectra can be pragmatic due to the n-*π*^*∗*^ transition.

Firstly, the MB dye molecules get adsorbed onto the surface of Ag-NPs. When Ag-NPs absorb incoming solar radiations (i.e., hv > Eg), electron-hole pairs are created in Ag-NPs. These photo-generated electron-hole pairs wander through the material and eventually reach the Ag surface. Similarly, the free radicals are designed when the holes in the valence band react with the surface molecules; for example, hydroxyl radicals (OH.) and superoxide anions (O_2_^−^) are formed when they react with the hydroxyl groups and H2O molecules present in the aqueous solution of MB dye. Concerning the conduction band, the photo-generated electrons combine with the O_2_ in air and aqueous solution of MB dye to form highly reactive species (OH. and O_2_^−^ radicals). These free radicals cause the degradation of MB dyes and release by-products such as water and CO2 [42, 43]. During photodegradation, the MB dye is converted to Leuco MB due to the destruction of azo bonds (-N=N-). Degradation efficiency of MB dye (%) was estimated by equation (3).

(3) $$\begin{array}{c} \frac{\left(D.E\right)\%=\left(C0-C\right)}{C0\times 100}, \end{array}$$

where C (mg/L) and C_0_ (mg/L) are the equilibrium and initial concentration of MB dye [44]. Degradation kinetic studies were used to estimate the photocatalytic degradation performance of biotreated Ag-NPs. The degradation kinetics were determined using the pseudo-first-order kinetics model, which can be characterized as follows:

(4) $$\begin{array}{c} -\ln\left(\frac{Ct}{C0}\right)=-kt, \end{array}$$

where *C*_t_ represents the temporal concentration of MB at time *t*, C_0_ represents the starting concentration of MB, *t* represents the degradation reaction time, and *k* represents the apparent photocatalytic degradation reaction rate constant. Degradation efficiency increases with an increase in adsorption time. With increasing photocatalyst and irradiation duration, the typical absorption of MB at 655 nm diminishes quickly. No additional absorption peaks rise during the process, indicating that the MB has completely degraded. Silver nanoparticles result in a degradation efficiency of 90% at the end of 120 minutes. Silver nanoparticles result in the degradation rate constants of 0.01533 min^−1^. Figure 8 shows the schematic representation of the photocatalytic activity of silver nanoparticles. As a result, the current investigation confirms that the produced Ag-NPs may exhibit high photostability, sustainability, and photo corrosive resistance during the photocatalytic destruction of MB dye when exposed to sunlight [45] (see Figure 10).

### 3.8. Morphological Stability of Ag Photocatalyst

Figure 11 shows the morphological stability of Ag-NPs after the photodegradation of MB dye molecules. TEM was castoff to determine the morphological stability of the regurgitated photocatalyst. The TEM photograph of the Ag-NPs confirms that no morphological changes have occurred after the degradation of MB. Under simulative visible-light irradiation, the as-prepared Ag-NPs demonstrate high photostability and reusability [46].

### 3.9. Antibacterial Activity

Figure 12 demonstrates the antibacterial activity of as-fabricated Ag-NPs. Ag-NPs are widely used in different biomedical applications due to their promising activity towards the inhibition of growth of microbial pathogens. The antibacterial efficacy of Ag-NPs was tested against *E. coli* and *S. aureus* bacterial pathogens. Ag-NPs displayed operative antibacterial activity towards both Gram-positive and Gram-negative bacteria. The antibacterial activity of Ag-NPs was maintained due to electrostatic interaction between positively charged Ag ions and negatively charged microbial cell surfaces, which allow them to interact with the bacterial cell wall and thereby resist the growth of bacteria [47].

Ag-NPs bind bacterial cell walls to disrupt the permeability and respiration, depending on the surface area available for interaction. Smaller particles with enhanced surface area allow more efficient penetration across cell walls than larger particles [48]. Consequently, the size and shape of fabricated Ag-NPs impact their antibacterial activity, and the effect of antibacterial activity increases when the size of NPs decreases. The antibacterial possessions of as-fabricated Ag-NPs eliminate or inactivate the harmful microorganisms in contaminated water. In comparison to other chemically synthesized Ag-NPs, the green Ag-NPs are ecologically safe and harmless due to the biologically reduced capping agents [49].  Figure 13 shows the plausible antibacterial mechanism of Ag-NPs.

### 3.10. Antifungal Activity

Figure 14 shows the antifungal activity of as-prepared green Ag-NPs. The antifungal activity of Ag-NPs was tested on *C. albicans.* Although the mechanism of Ag-NPs' fungicidal activity is not known, it is assumed that Ag-NPs prevent budding by forming holes on the fungal cell membranes, which ultimately prime to cell death [50]. Furthermore, the antibacterial activity of Ag-NPs has been attributed to the mediation of free radicals, which cause significant damage to the basic structure of DNA and proteins. Due to their smaller particle size, the NPs penetrate through the fungal cell membrane, fix to their functional groups, such as amino group, phosphorous, carboxyl group, and sulphur-containing substances, thereby inducing death of fungal cells. Release of Ag ions might also be the primary cause of the antifungal activity of Ag-NPs [51].

### 3.11. Anticancer Activity

The cytotoxic effect of Ag-NPs synthesized from bark extract of *Thespesia populnea* on the viability of SK-EML cancer cells was strong-minded by using MTT assay. Apoptosis is a primary therapeutic characteristic to treat cancer cells as it is avoided by cancer cells, which allows them to proliferate. Plant-based nanosized Ag-NPs are gaining importance in treating various cancers. To initiate apoptosis, two signalling pathways, for example, intrinsic and extrinsic pathways, are followed by cell. In malignant cells, programmed cell death is prompted by either damaging DNA or causing extreme cell stress [52]. Ag-NPs synthesized by bioactive fraction of *Pinus roxburghii* were found to have a cytotoxic effect against lungs and prostate cancer cells. The results showed that mitochondrial depolarization leads to DNA damage through intrinsic pathway. Cellular senescence of cancer cells is also triggered by an increase in reactive oxygen species (ROS), cell cycle arrest, and caspase-3 activation [53]. The Ag/Cu-NP alloy causes selective toxicity in breast cancer MCF-7 cells, suggesting that it might be used as a potential anticancer agent [54]. Aqueous extract of *Agaricus bisporus* fungus was used to biologically fabricate Ag-NPs. On MCF-7 breast cancer cells, Ag-NPs had a dose-dependent lethal impact with an LD_50_ (50 *μ*g/ml). Compared to the tumour group, mice with Ehrlich solid tumours treated with Ag-NPs and subjected to gamma radiation had dramatically better quality superoxide dismutase and catalase activity, decreased glutathione, and increased malondialdehyde and nitric oxide levels [55].

The MTT assay was employed to examine the anticancer activity of Ag-NPs by calculating the percentage of cell viability (living cells), and IC_50_ values were calculated for each cell line. Doxorubicin, an FDA-approved drug, was used as a positive control. The potential cytotoxicity of Ag-NPs against SK-MEL cells was concentration-dependent. At a dose of 12.5 and 50 *μ*g/mL, Ag-NPs produced 50% cytotoxicity against SK-MEL-28. The strongest inhibitory action was indicated by a lower IC_50_ value of 45.01 [56]. In SK-MEL cancer cells, with varying doses of the material, a dose-dependent decrease in cell viability was detected. The IC_50_ concentration was determined to be 45.01 *μ*g/mL with percentage viability of 78.95, as shown in Table 1.

#### 3.11.1. Morphological Study of Cancer Cells Treated with Ag-NPs

*Thespesia populnea* bark extract-mediated Ag-NPs were used to incubate melanoma cell lines at various concentrations.  Figure 15 shows the cytotoxic potential of as-prepared NPs through MTT assay. The morphology and viability of cancer cell lines were inspected by FLoid Cell Imaging Station. Ag-NPs-treated cells exhibited irregular structures, for example, roundness, stressed cells, cytoplasmic vacuoles, and larger cells; on the other hand, the normal cells showed regular structure with their nuclei (Figure 15).

#### 3.11.2. Mechanism of Anticancer Activity

The apoptosis of cancer cells begins with the stimulation of apoptotic proteins, followed by DNA damage, mitochondrial disintegration, and the development of an Apoptosome, which finally leads to cell shrinkage. Ag-NPs own anticancer properties which operate on specific target areas. According to recent findings, the Ag-NPs primarily function by increasing reactive oxygen species (ROS), a free radical by-product of cellular metabolism and necessary for maintaining cellular homeostasis. Moreover, the Ag-NPs are found to show oxidative stress as well as DNA damage through signal transduction pathways. The Ag-NPs-induced toxicity outperformed the production of intracellular ROS, which causes DNA, lipid, and protein damage.

## 4. Conclusion

The silver nanoparticles were fabricated by using *Thespesia populnea* bark extract as a reducing agent followed by characterization. The XRD pattern of as-prepared NPs demonstrates that the fabricated silver NPs have a face-centred cubic structure with 17-18 nm crystallite size. SEM analysis characterizes their agglomerated spherical shape. TEM investigation reveals the uniform distribution of spherical NPs. Ag-NPs showed a small bandgap, which implied their remarkable affinity towards absorption of visible light, making it a promising and appealing photocatalyst. Ag-NPs showed high photodegradation efficiency (up to 90%) and a rate constant of 0.01533/min. The hydroxyl radicals (^•^OH) were the main reactive oxygen species during the degradation of MB. Additionally, the as-synthesized photocatalysts showed better morphological stability as well as reusability. The heightened photocatalysis and degradation efficiency can be attributed to their smaller crystallite, particle size, surface aggregation with voids, strong optical absorption in the visible range, quick charge transfer, lower electron-hole recombination rate, and high oxidizing ability. In the near future, the as-prepared Ag-NPs might find their application as promising visible-light-driven photocatalyst for environmental remediation. Ag-NPs showed effective antibacterial, antifungal, and cytotoxic activities, with tests revealing an increase in cancer cell viability against SK-MEL cell lines.

## Figures and Tables

**Figure 1:** Synthesis of Ag-NPs using *Thespesia populnea* bark extract.

**Figure 2:** XRD spectra of Ag-NPs.

**Figure 3:** FTIR spectra of silver nanoparticles using *Thespesia populnea* bark extract.

**Figure 4:** UV-visible absorbance spectra of Ag-NPs.

**Figure 5:** UV-visible absorbance spectra after 4 months.

**Figure 6:** UV-visible absorbance spectra of Ag-NPs.

**Figure 7:** EDX spectra of Ag-NPs.

**Figure 8:** TEM image of Ag-NPs.

**Figure 9:** (a) Time-dependent UV-Vis absorbance spectra of MB dye degradation, (b) degradation efficiency, and (c) pseudo-first-order kinetics.

**Figure 10:** Plausible photocatalytic degradation mechanism of MB dye over Ag-NPs.

**Figure 11:** Morphological stability of silver nanoparticles after degradation of MB.

**Figure 12:** Antibacterial activity of silver nanoparticles.

**Figure 13:** Plausible antibacterial mechanism of Ag-NPs.

**Figure 14:** Antifungal activity of Ag-NPs.

**Figure 15:** Effect of Ag-NPs concentration on bacterial cell viability.

**Table 1:** Effect of Ag-NPs concentration on bacterial cell viability

Samples	Triplicate 1	Triplicate 2	Triplicate 3	Average
Control	0.602	0.584	0.596	0.594
12.5	0.481	0.466	0.46	0.469
50	0.331	0.342	0.353	0.342
Concentration (µg/ml)	Percentage viability			IC 50
12.5	78.95			45.01
50	57.57			

## Data Availability

No data were used to support this study.
